# Piano Teaching Knowledge Graph Construction Based on Cross-Media Data Analysis and Semantic Network

**DOI:** 10.1155/2022/5499593

**Published:** 2022-06-16

**Authors:** Han Li

**Affiliations:** Music and Dance College, Heze University, Shandong, Heze, China

## Abstract

With the rapid development of information technology and mobile Internet, digital image, text, audio, video, and other cross-media data are growing explosively, which has changed people's way of life and work. In view of the issues of negative studying effectivity and challenging attention of college students in the modern-day piano instructing process, this paper puts forward the application of knowledge Atlas technology in piano teaching and constructs a multimodal knowledge Atlas of piano teaching based on deep neural network, so as to make piano teaching more intelligent and improve students' learning efficiency and learning interest. How to realize the semantic association understanding of cross-media data is the core problem of cross-media semantic analysis. First, this paper introduces the basic rules of ontology construction and the basic method of establishing general knowledge graph are introduced. Then, taking the piano teaching content as an example, natural language sentences can be expressed and stored with cross-media data using semantic network. The mathematical understanding is extracted in accordance to the herbal language processing technology, and the entities are fused in accordance to the frequent semantic similarity detection between extraordinary entities, so as to decrease the redundancy and repetition fee of entities and the complexity of the graph. The fused new knowledge is processed according to the quality evaluation rules, the qualified part is added to the knowledge base, and then the above steps are iterated to update the database. The great overall performance of piano instructing understanding graph mannequin primarily based on semantic network is validated through experiments.

## 1. Introduction

With the speedy improvement of synthetic talent and people's interest to education, innovative teaching methods have attracted more and more attention. In college classroom, teachers' teaching method is no longer traditional blackboard writing, but transformed into multimedia teaching including text, courseware, video, voice, and other forms. However, the general framework of curriculum knowledge is mainly shown in the form of catalog of chapters in textbooks, while the small knowledge points are contained in the chapters and the relationship between knowledge points cannot be seen at a glance, which is not conducive to students' learning [1]. Therefore, how to effectively integrate the various forms of curriculum resources and better organize and present knowledge has become a research topic of great significance. In the teaching process of teachers, a variety of curriculum resources will be produced and exist in the form of text, audio, and so on [2]. Curriculum resources themselves have the characteristics of multimodal. At present, most of the resources of various modes exist and are used alone, and the curriculum resources between different modes produced in the classroom are rarely integrated to play a greater role. How to effectively organize and manage the curriculum knowledge, present the obscure knowledge in a more intuitive form, and help students learn more efficiently [3]. Therefore, constructing the knowledge graph of teaching is a particularly important research work.

The concept of knowledge graph has been proposed by Google since 2012. As the semantic knowledge base behind Google search engine, it is an advantageous structure of understanding agency and administration and a wonderful potential to resolve the above problems. Because of the intuitiveness and interpretability of understanding graph, it is extra and extra-utilized in exclusive vertical fields, such as finance, law, scientific therapy, and so on. For the field of education, as a multimodal knowledge base, curriculum includes text, audio, and other multimodal resources [4]. Different types of data depict rich semantic information, respectively, only constructing a single-text modal knowledge graph often that can only obtain some characteristics of cognitive objects, which are easy to bring certain limitations [5]. Multimodal curriculum expertise sketch can first be truly specific only if the semantic relationship between knowledge, efficaciously clear up the hassle of scattered and susceptible relevance of curriculum knowledge, enhance the deficiency of present information representation, information beginners to structure a right cognitive shape, and higher comb understanding [6]. At the same time, it can fully mobilize users' multiple senses to participate in learning and stimulate users' interest in learning. The design of knowledge graph can help users learn in an exploratory way, expand learning resources, support users to discover knowledge, and have a deep understanding of the content.

In this paper, taking the piano educating path as an example, this paper integrates the information from exceptional sources and structures, extracts the entities contained in the records and the semantic relationship between entities, constructs the multimodal curriculum know-how graph, and places ahead the building of piano instructing multimodal information graph based totally on deep neural network. On the one hand, the facts of elements are displayed in the shape of intuitive and clear information graph, which is conducive to the mastery of knowledge. On the exceptional hand, the multimodal curriculum statistics layout constructed in this paper makes the textual content material and speech modal curriculum property complement each other, realizes the integration of multimodal property and the reading route retrieval of knowledge elements at the bottom of the curriculum, and helps university college students analyze efficiently. The organizational shape of this paper is as follows.  Section 1 is the introduction, which introduces the heritage and magnitude of the topic, and introduces the lookup content material of this paper.  Section 2 is the associated work, discussing the lookup reputation at domestic and overseas and summarizing the associated work.  Section 3 is the theoretical foundation of setting up know-how graph primarily based on deep neural network, which normally introduces the simple theories associated with this paper. In Section 4, the parameter assessment scan and evaluation are carried out.  Section 5 is the precis and prospect. This section makes a complete precis of the techniques proposed in this paper and discusses the viable in addition lookup work in the future.

## 2. Related Work

The thinking of expertise graph is typically utilized to commercial enterprise situations such as Internet-oriented search, recommendation, and so on. Knowledge graph is divided into established understanding graph and vertical area understanding graph, and vertical domain knowledge graph emphasizes depth. As an effective knowledge organization model, knowledge graph has been widely used in e-commerce, biomedicine, law, sociology, education, and other fields. At present, some scholars are engaged in the research of multimodal knowledge graph, combined with deep neural network, and the main research of multimodal knowledge graph is as follows:

In the field of education, the knowledge graph can be used to analyze the development and research status of the discipline, explore the cooperative relationship between scholars, help scholars understand the discipline development trend, and quickly grasp the cutting-edge hot spots [7]. Some graph online courses from different providers, such as universities and MOOC, to the common space of concepts and predict the potential premise dependencies between concepts and courses. K-12edukg system can automatically build a knowledge graph for *K*-12 education discipline, use named entity recognition technology to extract educational concepts, and use data mining technology to identify the cognitive prerequisite relationship between educational concepts [8]. The literature suggests how to clearly present the internal structure of knowledge graph which is particularly important, and there are few relevant visualization studies at present [9]. The extracted entities and entity relationships are used to construct the graph of educational knowledge, and a visual analysis platform is constructed [10]. The literature suggests that the knowledge points in ball Cui should be divided into hierarchical structures according to the curriculum outline. Some scholars were organized to build the integration model of knowledge points and developed the large system into belonging relationship, related relationship, and prerequisite relationship [11]. Let students clearly understand this orderly relationship and follow-up relationship, form a link between the contents of chapters, form an organic rest between knowledge points, and finally let students truly master the course knowledge [12]. An American enterprise looks up the questioning of knowledge elements in the understanding of design and the relationship between records points, defines the studying direction thru the relationship between nodes, and edges in the expertise graph, units the precursor prerequisites for the understanding points, assigns a state, and recommends the subsequent gaining knowledge of course and content material for college students via students' studying facts labels, so as to dynamically regulate the getting to know format [13]. Through the constructed educational knowledge graph, the literature predicts and analyses the hot spots of examination, so as to help the users learn the target.

In addition, some scholars are committed to the research of adaptive learning and construct the teaching knowledge graph by aggregating the knowledge points at different levels of disciplines and students' learning data. In recent years, some knowledge graph education platforms have also been produced [14]. Students can find their own knowledge points through the knowledge points of the squirrel graph and learn them at the same time. Gaohu learning platform collects students' writing data, evaluates students' learning ability, granulates and structures knowledge points, traces the source after mining students' knowledge points defects, and systematically plans learning paths [15]. IFLYTEK platform of university of science and technology accurately pushes learning resources for students, forms a super wrong question book with clear logic, and realizes intelligent recommendation [16]. Generally speaking, most of the present instructional understanding graphs are K-12 simple instructional understanding graphs and the integration of online curriculum assets at the macrolevel. There is less-research work on the educational knowledge graphs of college students and the combing of the knowledge points at the bottom of the discipline [17]. At the same time, regardless of the resources generated in the network or in the classroom, the curriculum itself has the characteristics of a multimodality. With more and more research and development of multimodal knowledge graph technology, the construction of multimodal curriculum knowledge graph is particularly necessary and meaningful.

## 3. Construction of Knowledge Graph Based on Deep Neural Network

Deep neural community is the groundwork of deep learning, deep neural community simulates human talent for evaluation and mastering via nonstop multilayer nonlinear processing process, and combines low-level points to structure extra abstract high-level facets or attributes. Convolutional neural network and cyclic neural network are two kinds of network models commonly used. These two neural networks can extract feature information well, so they are widely used in various tasks [18]. Convolution neural network is a convolution of the information of some windows in a sequence. Therefore, it performs a full-size position in extracting neighborhood features, and cyclic neural community and long-term and momentary reminiscence community can manner sequence data well, so they are regularly used to extract the data of sequence information which includes text.

### 3.1. Convolutional Neural Network

Convolutional neural community is a feedforward neural community composed of one or extra convolution layers, pooling layers, and the full connectivity layer corresponding to the classical neural community at the top. Convolutional neural community can additionally be educated by way of the back-propagation algorithm delivered earlier; however, it wishes to study an awful lot fewer extremely good parameters than different normal deep feedforward neural networks, and the complexity of the mannequin is substantially reduced, so it can be skilled extra-effectively.

The overall performance of convolutional neural community in the subject of photograph attention and speech evaluation is needless to say higher than the ordinary deep neural community structure. It can be stated that this shape of convolution is mainly designed for gaining knowledge of two-dimensional statistics [19]. The community shape traits of weight sharing are very comparable to organic neural network. When the center of the community is multidimensional data, we can analyze the spatial correlation. At the equal time, the large-scale photo can additionally be at once at the center of the neural network. The end-to-end mannequin bypasses the operation of function extraction and facts compression in the regular algorithm [20]. Convolutional neural neighborhood makes use of the spatial correlation of center samples to limit the range of fantastic parameters to be observed in the coaching process. It is the first deep neural community algorithm that has been effectively educated and practiced in mainstream duties in many fields to gain amazing performance, which usually has advantages from three essential technical factors in the community structure:

#### 3.1.1. Partially Connected Network

In the standard deep neural network, the connection between the enter layer and the hidden layer is in full connection, that is to say, all neurons are connected in pairs. For a data set with a relatively small amount of single sample data, it is no problem to input the complete sample data into the network for operation. However, for data sets with large sample data, it will be very difficult to train a fully connected deep neural network because the parameters that need to be trained will increase exponentially compared with small sample data sets. According to the previous introduction, if the input layer has 10000 neurons and the second fully connected layer needs to output 100 features, the number of parameters to be learned is the product of these two values, that is, it will reach the order of millions. When the size of the input sample increases by *N* times, the number of input units will increase by *N* times, and the parameters to be trained in the network will also increase by *N* times. Accordingly, the training time of the whole network will be more than times slower.

Obviously, the explosive growth of the number of parameters of ordinary deep neural network is caused by the connection of all interlayer nodes. The most direct way to remedy this trouble is to restrict the connection between the nodes of the enter layer and the hidden layer, and construct a subset of input neural elements according to a certain strategy to connect with the corresponding single-hidden layer neuron [21]. For example, a large complete picture is divided into small adjacent areas, and such a local picture is used to connect the neurons of the hidden layer. For different enter forms, such as the audio sign and lyrics textual content for this study, the nearby vicinity linked with the hidden layer unit can be chosen in accordance to the traits of the sequence information, such as the sign or textual content in some nonstop quick time period. In fact, biologists have found that in the structure of human visual system, neurons in the visual cortex only receive local stimulation in some specific areas Figure 1.

#### 3.1.2. Convolution

When a natural image is divided into several small blocks, although the high-level semantics expressed by these small areas may not be complete, they are still a complete image data. In other words, from the perspective of data attributes and statistical characteristics, one part of an image is independent and the same as other parts [22]. Applying this idea to statistical machine learning, it can be considered that the method of learning features in one subregion of an image can also be used in another subregion, which means that all subregions of an image can share the same feature learning method. Basic model of convolutional neural network is shown in Figure 1.

### 3.2. Cyclic Neural Network

In addition to the input of current information, each neuron of cyclic neural network also has previously generated memory information, which retains the sequence-dependent type. Many tasks need to process sequence data. For example, image subtitles, speech synthesis, and music generation all need model generated sequence data. In other fields, such as video analysis, music information retrieval and time series prediction, the enter and output of the mannequin are required to be sequence data, such as computing device translation and man-machine dialogue. RNN mannequin can be used to method sequence data. RNN carries a giant variety of parameters and is hard to train, so there is a sequence of optimization of RNN, such as community structure, answer algorithm, and parallelization.

Through a series of point-to-point scaling transformations, the number of Fisher information conditions of the network is improved, and various adverse effects caused by the symmetry of the weight space of the deep neural network on the neural network training are solved, so as to improve the training speed of the deep neural network. Let *C*_*k*_(*i*, *j*) represent the expected value of the gradient square of the weight parameter *w*_*k*_(*i*, *j*) on the training data set in layer *k*, that is,

(1) $$\begin{array}{c} C_{k}\left(i,j\right)=\frac{\partial L}{\partial w_{k}\left(i,j\right)},\\ C_{k}^{2}\left(i,j\right)={\left(\sigma_{k-1}\left(j\right)\frac{\partial L}{\partial w_{k}\left(i,j\right)}\right)}^{2}. \end{array}$$

In order to calculate the approximate learning rate of a weight parameter, the following formula is formed:

(2) $$\begin{array}{c} \overset{\wedge }{C_{k}^{2}}\left(i,j\right)=\frac{C_{k}^{2}\left(i,j\right)}{{\left\|w_{k}\right\|}^{2}}. \end{array}$$

In the deep neural network, this effect is nonlinear. It is required that the average learning rate of weight parameters in all columns of the weight matrix is roughly the same, as shown in the following formula:

(3) $$\begin{array}{c} \overset{\wedge }{C_{k}^{2}}\left(:,j\right)=\frac{\sum \overset{\wedge }{C_{k}^{2}}\left(i,j\right)}{\left[\sigma_{k-1}{\left(j\right)}^{2}{\left\|y_{k}\right\|}^{2}\right.}. \end{array}$$

When propagating forward, the preactivation value can be expressed by the following recursive relationship:

(4) $$\begin{array}{c} h_{j}^{l+1}\left(\alpha \right)=\sum \left(X_{i}^{l}\left(\alpha +\beta \right)\right)\omega_{ij}^{l+1}\left(\beta \right)+b_{j}^{l+1}. \end{array}$$

Considering the calculation formula of weight parameter gradient of layer *l*:

(5) $$\begin{array}{c} \frac{\partial E\left(X^{L},y\right)}{\partial \omega_{ij}^{l}\left(\beta \right)}=\sum \frac{\partial X_{t}^{l}\left(\alpha \right)}{\partial \omega_{ij}^{l}\left(\beta \right)}\frac{\partial X_{k}^{L}\left(\gamma \right)}{\partial X_{t}^{l}\left(\alpha \right)}\frac{\partial E\left(X^{L},y\right)}{\partial X_{k}^{L}\left(\gamma \right)}. \end{array}$$

For the deep fully connected residual network, after simple derivation, the Jacobian matrix of its output to the input of layer *l* can be expressed as follows:

(6) $$\begin{array}{c} \frac{\partial X_{i}^{L}}{\partial X_{k}^{l}}={\left[\prod_{i=l+1}^{L}\left(D^{i}W^{i}+1\right)\right]}_{ik}. \end{array}$$

Each convolution kernel and each channel perform convolution operation independently, so the output of the convolution layer has the following block matrix form for the input Jacobian matrix:

(7) $$\begin{array}{c} \frac{\partial Y}{\partial X}={\left[\frac{\partial \left(Y_{1\times n}\right)}{\partial X},\ldots ,\frac{\partial \left(Y_{i\times n}\right)}{\partial X},\ldots ,\frac{\partial \left(Y_{i\times n}\right)}{\partial X}\right]}^{T}. \end{array}$$

The recurrent neural network obtains a unique network structure by adding a self-connected hidden layer across time points, which makes it master the ability of explicit modeling of time. After increasing the shape of the recurrent neural community in accordance to the time point, it can be observed that the remarks of the hidden layer are output now not solely to the subsequent layer; however, additionally to the neurons of the identical hidden layer at the subsequent time point. In other words, the hidden-layer node of recurrent neural community will get hold of the center of the contemporary time factor and the output of the hidden layer of the preceding time factor at the equal time. In order to adapt to this special twin, enter structure, the hidden-layer nodes of the recurrent neural community have reminiscence storage characteristics, and the inner reminiscence content material will be up to date in accordance to the replacing of the enter data. The last output of recurrent neural community is bought by means of integrating the enter of the contemporary time factor and the information of the preceding time factor saved with the aid of the hidden-layer node [23].

### 3.3. Construction of Multimodal Knowledge Atlas

In the context of big data technology, the Internet has accumulated huge amounts of data and information. In order to embody its utilization value, we must eliminate the dross and extract the essence. Therefore, knowledge databases in all walks of life have been established. These out-of-order information resources have been organized into basic knowledge base for subsequent production practice, scientific research and development, and practical application. In a broad definition, knowledge base is a management tool of structured data, which is used to obtain knowledge information in a certain field and is suitable for subsequent application research [24]. According to the description in relevant literature, the definition of knowledge base is divided into two categories: first, in the field of information science and enterprise management, knowledge base refers to a kind of document base, which specially stores various data documents, case files, program reports, and other contents. Second, in the field of control engineering and computer science, knowledge base refers to a database with clear hierarchy, clear structure, and modular management.

The top-level design, that is, the conceptual pattern layer, is generally considered first in constructing most knowledge graphs, in other words, the data organization of knowledge base. Since it is the knowledge graph of subdivided fields or the knowledge graph of general fields, it needs relevant data as support. If you want to selectively collect target data in these large amounts of data, you need to formulate corresponding rules and standards, and its source is the data model [25]. Therefore, the definition of conceptual mannequin is genuinely to formulate a set of guidelines that take impact in this expertise system. It is required that the information format solely accepts and consists of the required goal information types. Determining the data model according to the characteristics of the knowledge graph is equivalent to determining the scope of the data collected by the knowledge graph. The construction process of knowledge graph is a continuous cycle and iterative task with good expansibility. Each update cycle has four main processes: knowledge extraction, knowledge storage, knowledge fusion, and knowledge calculation. As shown in Figure 2.

Because this paper has a wide range of data sources and rich data modes, after in-depth study of the construction requirements and construction technology of multimodal graph, this paper selects relevant fields to construct the vertical domain multimodal knowledge graph [26]. The data sources are encyclopedia websites and related websites containing text, pictures, and videos. Some key technologies in the construction of multimodal knowledge graph are comprehensively used to study the construction of multimodal knowledge graph. The relevant technical methods are shown in Figure 3.

The methods in the process of constructing multimodal knowledge Atlas include data acquisition and processing, schema construction, multimodal knowledge extraction, multimodal knowledge fusion, Atlas visualization, and Atlas application. Among them, the methods used in multimodal knowledge fusion include calculating similarity, label alignment, and data link. If these multisource heterogeneous data are directly used, the subsequent construction and application will be greatly affected due to the different organization and composition of the data, and there are some unavailable fragment data [27]. Therefore, these multisource heterogeneous data must be preprocessed first to ensure the basic correctness of the subsequent process.

## 4. Results and Analysis

In the procedure of mannequin training, there are two vital parameters: mastering price and dropout value. If gaining knowledge of charge is too large, the mannequin will converge too quick and can also exceed the superior value. If the mastering price is too small, the mannequin will converge too slowly, have an effect on the coaching efficiency, and even motive the mannequin to fail to converge. Therefore, this paper provides the comparative experiments of gaining knowledge of charge and dropout fee to discover the mannequin with the exceptional effect.

### 4.1. Comparative Analysis of Learning Rate

First, through continuously adjusting the getting-to-know price and evaluating the mannequin results when the studying charge is 0.01 and 0.001, respectively, it is found that the *F*1 value when the learning rate is 0.01 is higher than that when the learning rate is 0.01, and the effect is better. Therefore, the learning rate used in this paper is 0.01.  Figure 4 is a comparison diagram of model recognition corresponding to two learning rates.

At the equal time, dropout technique can be used to keep away from over becoming phenomenon in mannequin training. Dropout is to make a neuron in accordance to a sure likelihood in the procedure of ahead propagation *Р.* Temporarily give up the work so that the mannequin has improved generalization ability, does now not remember too a great deal on some neighborhood features, and achieves the impact of regularization to a sure extent. When the mastering fee is 0.01, dropout is set to 0.1 and 0.5, respectively. It can be considered that the hole between the two is no longer large. As dropout is more secure when dropout is 0.5, this paper subsequently adopts the case that dropout fee is 0.5. The loss cost decreases progressively with the increase of the variety of epoch of new release rounds, and after 10 rounds of iteration, the loss decreases to a smaller fee and is pretty stable. Through the evaluation take a look at the above parameters, the mannequin will be getting to know the charge of 0.01 and dropout cost of 0.5 is sooner or later selected, as proven in Figure 5.

### 4.2. Comparative Analysis with Other Models

This paper compares three companies of entity focus methods, which are based totally on CNN + BILSTM-CRF model, BILSTM-CRF mannequin, and information graph mannequin primarily based on deep neural network. Each mannequin has been skilled for 15 rounds. The contrast of experimental outcomes is proven in Figure 6.

It can be viewed from the experimental consequences that every mannequin can attain a positive impact of entity recognition. Among them, the accuracy and recall of CNN + BILSTM–CRF mannequin are expanded via 0.3% and 3.6%, respectively, on the foundation of BILSTM-CRF model. It is considered that the impact of CNN + BILSTM–CRF mannequin in this paper is higher than that of BILSTM–CRF model. It indicates that the aggregate of CNN and BILSTM can successfully use nearby and world records to attain extra whole textual content features, which make the mannequin extra-correct and can reap higher named entity cognizance effect. After including the area dictionary, the F1 cost has expanded to 2.6% on the foundation of CNN + BILSTM–CRF model, which is considered to assist in addition to enhancing the impact of the model. In conclusion, the know-how graph mannequin primarily based on deep neural community proposed in this paper can reap desirable consequences in entity recognition and can substantially enhance the impact of entity attention to a sure extent after the introduction of area dictionary. This paper additionally makes use of this mannequin to complete the entity prediction of unmarked textual content data, so as to make certain the entity statistics have a first-rate understanding of the graph.

### 4.3. Analysis of Piano Teaching Effect

Generating experimental facts from piano song information set, thinking about that emotion classification is the most frequent venture in the discipline of herbal language processing, and the assignment of this test is the automated labeling of emotion tags. In the process of building the automatic annotation model, many parameters need to be explored and adjusted according to the experimental results. As cited above, in accordance to the commentary of phrase segmentation results, it is discovered that the Chinese phrase segmentation algorithm does not function properly in the extraordinary corpus of lyrics; however, whether or not this hassle will without a doubt have an effect on the labeling impact, nevertheless, wants experimental verification, and then is how to pick the dimension of phrase embedding. According to the previous introduction to word vectors, the feature dimension of each word can be set to any value. If the chosen dimension is too small, the phrase vector is now not ample to characterize all the records of the text. If the chosen dimension is too large, the illustration of the text will be too sparse, and the getting-to-know price of the deep neural network will be reduced. The shape and amazing parameter optimization of deep neural community rely on the comments of the experimental process.

First, the optimal minimum unit in text preprocessing is verified. In this experiment, four schemes were selected: single word, word segmentation vocabulary, bigram, and trigram. Among them, two characters' words and three characters words are very common concepts in the field of natural language, which refers to taking two or three adjacent Chinese characters as independent units, and the step length is one Chinese character. On the optimal network proposed in this chapter, experiments are carried out for different schemes. After determining the single word as the minimum text-processing unit, the word vector generation tool word2vec is used to generate the word vector of each word based on cow model. For different word vector dimensions, a series of experiments are carried out on the optimal network proposed in this chapter, and the results are shown in Figure 7.

As can be seen from Figure 7, the dictionary capacity increases significantly with the change of processing unit, which is also in line with the analysis. Annotation mannequin indications exhibit that the impact of phrase vector as enter function is the best, and all four indications are notably greater than different sorts of enter features. The impact of two-character phrases as the minimal processing unit is additionally higher than that after phrase segmentation, which suggests that the contemporary Chinese phrase segmentation equipment cannot deal with the lyrics textual content well. The impact of three-character phrases is the worst. It is likely that when the dictionary dimension is too large, the text representation is too sparse. With the increase of word vector dimension, the annotation effect of the model continues to improve, but when it reaches the critical point of 600 dimension, the annotation effect of continuing to increase dimension is almost unchanged.

Experiments on different deep learning algorithms are carried out on the self-help data set. At the theoretical level, convolutional neural network is a hierarchical structure, while cyclic neural network is a sequence structure. In practice, all input samples of the convolutional neural network must have the same size of characteristic matrix, and cyclic neural network can accept the input of variable length sequence. In the previous experiment, according to the statistics of the length of lyrics, 400 words were selected as the upper limit of length. Only 400 words are reserved for lyrics with more than 400 words, and zero is filled after the characteristic matrix for lyrics with less than 400 words. The cyclic neural network can ensure that all samples input a complete text sequence. For more objective comparison, the upper limit of the lyrics text in the following experiment is set to 800 words, so as to highlight the characteristics that the cyclic neural network can include more original information without noise.

Figure 8 shows the performance of three different deep neural networks in the task of automatic music annotation based on lyrics. In terms of various indicators, convolutional neural network still performs better, which is also in line with the mainstream view that convolutional neural network is better than cyclic neural network in classification tasks in academic circles. It can be seen that in fact, the small change of convolution window size has no significant effect on the experimental effect.

## 5. Conclusion

This paper applies the information graph to piano teaching, takes the challenge of understanding factors as the entity, extracts attribute facts and multimedia sources from instructing materials, syllabus and network, and constructs the issue multimodal expertise graph. Based on the multimodal understanding graph, instructors can raise out greater multimodal sensible schoolroom teaching. In addition, information factor retrieval and visualization based totally on Atlas, wise lecture room teaching, customized studying, and instructing software can help instructors in cantered teaching. According to the getting-to-know state of affairs of every student, exceptional comparison outcomes are given to understand the actual customized self-sustaining learning. This paper places ahead a graph mannequin of piano instructing track understanding primarily based on deep neural network and introduces the motives for selecting phrase vector as textual content illustration and convolution neural community as community structure. Through comparative experiments, it is proved that the prediction stop end result of the piano instructing model primarily is based definitely on deep gaining expertise of is simply greater than the preferred multilabel classification algorithm, and in a similar way explores the impact of the neighborhood form and the adjustment of the specific parameters of the mannequin on the prediction effect.

## Figures and Tables

**Figure 1:** Basic model of convolutional neural network.

**Figure 2:** Frame diagram of knowledge graph construction.

**Figure 3:** Technical route of multimodal knowledge Atlas.

**Figure 4:** Comparative analysis of model renderings.

**Figure 5:** Comparison diagram of model effect when dropout value is determined.

**Figure 6:** Analysis of experimental results of different models.

**Figure 7:** Relationship between note length, vector dimension, and model effect.

**Figure 8:** Relationship between network structure and model effect.

## Data Availability

The data used to support the findings of this study are included within the article.

## References

[1] Matassi M., Boczkowski P. (2021). An agenda for comparative social media studies: the value of understanding practices from cross-national, cross-media, and cross-platform perspectives. *International Journal of Communication*.

[2] Li A., Du J., Kou F., Mingying X., Yang J. (2022). Scientific and technological information oriented semantics-adversarial and media-adversarial cross-media retrieval. https://arxiv.org/abs/2203.08615.

[3] Huang S. M., Ma L. G. (2022). Research on mixed teaching evaluation system based on deep learning [J]. *Journal of Gansu Radio and Television University*.

[4] Palomo B., Sedano J. (2021). Cross-media alliances to stop disinformation: a real solution?. *Media and Communication*.

[5] Wu H. J. (2021). Construction and application of personalized MOOC course based on multimodal knowledge atlas [J]. *Henan University*.

[6] Maulud D. H., Zeebaree S. R. M., Jacksi K., Mohammed A. M. S. (2021). State of art for semantic analysis of natural language processing. *Qubahan Academic Journal*.

[7] Du X. R., Yang H. Q. (2021). Teaching practice and thinking of supervised learning based on deep network. *Computer Education*.

[8] Huang Y. K., Liang M. Y., Wang X. X., Chen Z., Cao X. W. (2021). Multi person classroom behavior recognition in classroom teaching video based on deep spatiotemporal residual convolution neural network. *Computer Applications*.

[9] Ruan L., Wen S. S., Niu Y. M. (2021). Deep neural network visualization based on interpretable basis decomposition and knowledge graph. *Journal of Computer Science*.

[10] Zhou C. H., Wang H., Wang C. S. (2021). Research on geoscience knowledge graph in the era of big data. *Chinese Science: Earth Science*.

[11] Huang C. (2021). On music classroom teaching strategy based on deep learning. *MusicWorld*.

[12] Zhu J. C., Chen G., Xiang H., Li Z. C., Wu K. C. (2020). Student portrait model of hybrid teaching based on deep neural network. *Information Technology and Information Technology*.

[13] Lin X. C. (2020). Teaching design and exploration based on deep learning. *Scientific Consultation*.

[14] Hu H. Y. (2020). Life experience teaching: promoting deep participation in music learning. *Northern Music*.

[15] Yang C. N. (2020). “Three ingenious uses” in teaching to build a music classroom of deep learning. *Voice of the Yellow River*.

[16] Lin J. H., Mo Q., Zhou J. J., Mo S. Y., Xie X. X. (2019). Action teaching platform based on deep convolution neural network. *Digital Technology and Application*.

[17] Li Z. X., He F. Z., Liu A. (2019). Construction and application of multimodal teaching knowledge atlas. *Fujian Computer*.

[18] Ma J. Y. (2019). Music classroom towards deep learning - taking music appreciation teaching in senior high school as an example. *China Music Education*.

[19] Li Y. Y., Zhang X. L., Li X., Du J. (2019). Construction and innovative application of subject knowledge graph for wisdom education. *Research on Audio Visual Education*.

[20] Gao B. (2018). High school music teaching strategy from the perspective of deep learning. *Northern Music*.

[21] Xiong H. X., Yang Z. R., Jiang W. X. (2019). Research on semantic correlation of multimodal data in the construction of cross media knowledge graph. *Information Theory and Practice*.

[22] Liu J. (2018). On school music teaching from the perspective of deep learning [J]. *Contemporary Education and Culture*.

[23] Li R. F., Chen J. J., Zhou Y. Q., Wang X. J., Zhong Y. X. (2015). Discussion on the teaching of convolutional neural network in deep learning. *Computer Education*.

[24] Pan J. Z., Calvanese D., Eiter T., Yuting Z. (2017). Understanding author intentions: test driven knowledge graph construction. *Springer International Publishing*.

[25] Abu-Salih B., Al-Tawil M., Aljarah I., Amin B. (2021). Relational learning analysis of social politics using knowledge graph embedding. *Data Mining and Knowledge Discovery*.

[26] Akay A., Dragomir A., Erlandsson B. E. (2015). Network-based modeling and intelligent data mining of social media for improving care. *IEEE Journal of Biomedical & Health Informatics*.

[27] Lim S., Berry F. S., Lee K. H. (2015). Stakeholders in the same bed with different dreams: semantic network analysis of issue interpretation in risk policy related to mad cow disease. *Journal of Public Administration Research and Theory*.

